The article "lncRNA MIR4435-2HG Accelerates the Development of Bladder Cancer through Enhancing IQGAP3 and CDCA5 Expression" was retracted in 2024. Reasons: signs of a paper mill; suspected computer-generated content; unreliable results or conclusions; concerns about the data.

# lncRNA MIR4435-2HG Accelerates the Development of Bladder Cancer through Enhancing IQGAP3 and CDCA5 Expression

**DOI:** 10.1155/2022/3858249

**Published:** 2022-08-12

**Authors:** Tao Yang, Yan Li, Gang Wang, Liuxiong Guo, Fuzhen Sun, Shoubin Li, Xinna Deng, Junjiang Liu

**Affiliations:** ^1^Department of Urology, Hebei Provincial People's Hospital, Shijiazhuang, 050000 Hebei, China; ^2^Department of Hematology, Hebei Provincial People's Hospital, Shijiazhuang, 050000 Hebei, China; ^3^Fourth Department of Oncology, Hebei Provincial People's Hospital, Shijiazhuang, 050000 Hebei, China

## Abstract

**Background:**

Bladder cancer (BCa) is one of the most prevalent cancers occurring in the urinary system. Long noncoding RNAs (lncRNAs), in recent years, have emerged as crucial regulators in various biological processes of tumors.

**Aim:**

To identify the role of MIR4435-2 host gene (MIR4435-2HG) and uncover its molecular mechanism in BCa.

**Methods:**

Firstly, quantitative real-time PCR (RT-qPCR) analysis was used to examine MIR4435-2HG expression in BCa cells. Cell Counting Kit-8 (CCK-8), 5-ethynyl-2′-deoxyuridine (EdU), wound healing, and transwell assays were implemented to identify the role of MIR4435-2HG in BCa. RNA-binding protein immunoprecipitation (RIP), RNA pull down, and luciferase reporter assays were applied to explore the potential mechanism of MIR4435-2HG in BCa.

**Results:**

MIR4435-2HG was highly expressed in BCa. Moreover, MIR4435-2HG silencing abrogated BCa cell proliferation, migration, and invasion. In terms of underlying mechanism, MIR44352HG acted as a microRNA-2467-3p (miR-2467-3p) sponge to control the expression of IQ motif containing GTPase activating protein 3 (IQGAP3) and cell division cycle associated 5 (CDCA5), resulting in activation of the rat sarcoma virus (Ras)/rapidly accelerated fibrosarcoma (Raf)/mitogen-activated protein kinase (MEK)/extracellular signal-regulated kinase (ERK) and PI3K/AKT/mTOR signaling pathways.

**Conclusion:**

MIR4435-2HG involves in the progression of BCa, which might provide novel insights for BCa treatment.

## 1. Introduction

Bladder cancer (BCa) is defined as a type of malignancy in which certain cells become abnormal and multiple without control in the bladder. It is one of the most common cancers of the genitourinary tract and a leading cause of morbidity and mortality [1]. Epidemiologic studies have indicated that cigarette smoking and occupational exposures are major risk factors for the occurrence of BCa [2]. Up to date, the management of BCa remains challenging and complicated due to its heterogeneity [3]. Therefore, surgery, radiation, and chemotherapy are still considered as main therapeutic strategies [4]. Accumulating evidence has demonstrated that emerging biomarkers may help to promote the early detection and diagnosis of BCa [5]. Hence, it is urgent to explore novel molecular markers to improve the therapeutic effect for BCa patients.

The article "lncRNA MIR4435-2HG Accelerates the Development of Bladder Cancer through Enhancing IQGAP3 and CDCA5 Expression" was retracted in 2024. Reasons: signs of a paper mill; suspected computer-generated content; unreliable results or conclusions; concerns about the data.

It is widely acknowledged that long noncoding RNAs (lncRNAs) occupy a vital position in regulating a variety of cellular processes of cancers through various mechanisms [6]. For example, Shang et al. have manifested that PVT1 plays an oncogenic role in colorectal cancer through interaction with miR-214-3p [7]. Wang et al. have demonstrated that UCA1 hampers tumor growth in esophageal squamous cell carcinoma via modulation of the Wnt signaling pathway [8]. Ding et al. have revealed that MIF-AS1 suppresses breast cancer progression via competing endogenous RNA (ceRNA) mode [9]. Previous studies have reported that ceRNA refers to a class of RNA functioning as miRNA sponges to regulate messenger (mRNA) expression, which affects tumor development [10]. Moreover, dysregulation of lncRNAs has also been suggested to be associated with the pathogenesis of BCa [11]. For example, Zhan et al. have illustrated that SOX2OT enhances cell stemness in BCa through upregulating SOX2 [12]. Li et al. have proved that MAFG-AS1 accelerates BCa development via the miR-143-3p/COX-2 axis [13]. Wu et al. have declared that ZEB2-AS1 induces the occurrence of BCa by serving as a sponge for miR-27b [14].

MIR4435-2 host gene (MIR4435-2HG) is affiliated with the lncRNA class. lncRNA MIR4435-2HG has been reported to affect multiple cancers, including gastric cancer, hepatocellular carcinoma, and ovarian carcinoma [15–17], and all findings testify the oncogenic role of MIR4435-2HG in tumors. But its function in BCa remains to be unearthed. Some reports have uncovered the downstream molecular mechanism of MIR4435-2HG. For instance, MIR4435-2HG triggers tumor progression via targeting miR-128-3p to modulate CKD14 expression in ovarian cancer [18]. MIR4435-2HG facilitates tumor progression of cervical cancer cells via the miR-128-3p/MSI2 axis [19]. In addition, MIR4435-2HG promotes the aggressiveness of liver cancer cells via the miR-136-5p/B3GNT5 axis. Here, we intended to explore the MIR4435-2HG-mediated ceRNA network in BCa.

In this research, we intended to explore the investigation into the role and regulation mechanism of MIR4435-2HG in BCa.

## 2. Materials and Methods

### 2.1. Cell Culture

BCa cell lines (T24, HT-1197, HT-1376, and 5637) and normal cell line (SV-HUC-1) were all provided by American Type Culture Collection (Manassas, VA). T24 cell line was cultured in McCoy's 5a Medium, HT-1197 and HT-1376 cell lines both in Eagle's Minimum Essential Medium, 5637 cell line in RPMI-1640 Medium, and SV-HUC-1 in F-12K Medium. All mediums were added with 10% fetal bovine serum (Gibco) for cell culture at 37°C in 5% CO_2_.

The article "lncRNA MIR4435-2HG Accelerates the Development of Bladder Cancer through Enhancing IQGAP3 and CDCA5 Expression" was retracted in 2024. Reasons: signs of a paper mill; suspected computer-generated content; unreliable results or conclusions; concerns about the data.

### 2.2. Plasmid Transfection

Short hairpin RNAs (shRNAs) against MIR4435-2HG, IQGAP3, or CDCA5, as well as their respective controls, were all generated by Genechem (Shanghai, China) and used for gene silencing. IQGAP3 or CDCA5 was overexpressed by inserting the sequence of IQGAP3 or CDCA5 into pcDNA3.1 vectors (Invitrogen, Carlsbad, CA). miR-2467-3p mimics/inhibitor and corresponding negative controls were all supplied by RiboBio (Shanghai, China). Transfection of 2 *μ*L plasmids (knockdown or overexpression vectors: 0.8 *μ*g/50 *μ*L; miR-2467-3p mimics/inhibitor: a final concentration of 100 nM) into BCa cells in a 24-well format was conducted utilizing 1 *μ*L Lipofectamine 3000 (Invitrogen).

### 2.3. Quantitative Real-Time PCR (RT-qPCR) Analysis

RT-qPCR was performed as previously described [20]. Using TRIzol Reagent (Invitrogen), total RNA was extracted and complementary DNA (cDNA) was synthesized by RevertAid First Strand cDNA Synthesis Kit (Thermo Fisher Scientific, Rockford, IL). To evaluate the expression of genes, PCR was conducted utilizing SYBR Green PCR Master Mix (Applied Biosystems, Foster City, CA). Gene expression level was calculated as per the 2^-*ΔΔ*Ct^ method, normalized to the expression of endogenous control (GAPDH or U6). The experiment was independently done in triplicate. Primers used for RT-qPCR are reported in Supplementary Table 1.

### 2.4. Cell Counting Kit-8 (CCK-8) Assay

BCa cells were placed into 96-well plates at a density of 5 × 10^3^ cells per well. This assay was performed as previously described. After 24 h, 48 h, and 72 h of transfection, each well was added with CCK-8 reagent. Subsequent to 2 h of incubation, the absorbance at 450 nm was measured. The experiment was independently conducted in triplicate.

### 2.5. 5-Ethynyl-2′-deoxyuridine (EdU) Staining Assay

EdU staining assay was implemented as previously described [21]. BCa cells were placed on sterile coverslips in 96-well plates (5 × 10^4^ cells per well). Cells were incubated with EdU staining kit (RiboBio) and treated in DAPI staining solution for 5 min. Cell proliferation was observed under an Olympus fluorescence microscope (Tokyo, Japan). The assay was independently carried out in triplicate.

### 2.6. Wound Healing Assay

Wound healing assay was done as previously described [22]. A total of 3 × 10^3^ cells were inoculated into 6-well plates and cultured in medium with no serum for 24 h at 37°C. A pipette tip was used to make a straight scratch when cells reached 80% confluence. Afterwards, BCa cells were subjected to another 24 h of incubation. The scratches were monitored and recorded at 0 and 24 h. The assay was performed in triplicate. Wound areas were analyzed by ImageJ software.

The article "lncRNA MIR4435-2HG Accelerates the Development of Bladder Cancer through Enhancing IQGAP3 and CDCA5 Expression" was retracted in 2024. Reasons: signs of a paper mill; suspected computer-generated content; unreliable results or conclusions; concerns about the data.

### 2.7. Transwell Assay

Transwell migration or invasion assay was carried out by using a 24-well transwell chamber (Corning), with Matrigel (BD Bioscience) precoating only for invasion assay. Transfected BCa cells (8 × 10^3^~3.6 × 10^4^) were placed into the upper chamber with addition of serum-free medium. Complete culture medium was put into the lower chamber. Subsequent to 24 h of incubation, cells were fixed in methanol. Subsequently, 0.1% crystal violet was used to stain the migrated or invaded cells for counting. The experiment was independently executed in triplicate. Transwell migration and Matrigel invasion assays were performed as previously described [23].

### 2.8. Subcellular Fractionation

Isolation of cytoplasmic-nuclear RNA was conducted as previously described [24]. Utilizing PARIS™ Kit (Ambion, Austin, TX), cytoplasmic and nuclear fractions were separated followed by RNA quantification by RT-qPCR. In this assay, GAPDH or U6 was regarded as cytoplasmic or nuclear control individually. The assay was independently carried out in triplicate.

### 2.9. Fluorescent In Situ Hybridization (FISH)

MIR4435-2HG-specific RNA FISH probe was procured from RiboBio for cellular analysis, in light of the instruction of supplier. BCa cells went through incubation with FISH probe in hybridization buffer, then treated with DAPI staining reagent. Images were acquired using an Olympus fluorescent microscope. The assay was independently carried out in triplicate.

### 2.10. RNA Pull-Down Assay

RNA pull-down assay was executed as previously described [25]. In a word, BCa cells (1 × 10^7^) were treated with biotinylated MIR4435-2HG probe (Sigma-Aldrich, St. Louis, MO), followed by addition of magnetic beads (Millipore, Bedford, MA). The pull downs collected by magnetic beads were purified for PCR analysis. The experiment was performed in triplicate.

### 2.11. RNA-Binding Protein Immunoprecipitation (RIP)

RIP assay was conducted as previously described [26]. In accordance with the user guide, Magna RIP RNA-Binding Protein Immunoprecipitation Kit (Millipore) was employed for RIP assay. Cell lysates were incubated with Anti-Ago2 antibody (~1.5 mg/mL; Sigma-Aldrich) and anti-IgG antibody (2.38 mg/mL; Invitrogen) which were used for immunoprecipitation. Subsequently, the RNA was extracted from immunoprecipitates for RT-qPCR. The experiment was performed in triplicate.

### 2.12. Luciferase Reporter Assay

The wild-type (Wt) or mutant-type (Mut) sequence of MIR4435-2HG full-length, IQGAP3, or CDCA5 fragments covering miR-2467-3p binding sites was inserted into pmirGLO dual-luciferase vector for the construction of pmirGLO-MIR4435-2HG-Wt/Mut, pmirGLO-IQGAP3 3′-UTR-Wt/Mut, and pmirGLO-CDCA5 3′-UTR-Wt/Mut individually. After that, the reporter construct was cotransfected with control mimics or miR-2467-3p mimics (a final concentration: 100 nM) into BCa cells. Eventually, dual-luciferase reporter assay system (Promega) was applied to detect the luciferase activity. Luciferase reporter assay was conducted and analyzed as previously described [25]. The experiment was executed in triplicate.

The article "lncRNA MIR4435-2HG Accelerates the Development of Bladder Cancer through Enhancing IQGAP3 and CDCA5 Expression" was retracted in 2024. Reasons: signs of a paper mill; suspected computer-generated content; unreliable results or conclusions; concerns about the data.

### 2.13. Western Blot Analysis

Western blot was performed as previously described [20]. Firstly, protein samples were separated and shifted onto PVDF membranes (Millipore, Billerica, MA). Subsequent to sealing with nonfat milk, the membranes were subjected to overnight incubation at 4°C with the following primary antibodies against IQGAP3 (1.7 mg/mL, Invitrogen), CDCA5 (0.5 mg/mL, Invitrogen), EGFR (1 mg/mL, Sigma-Aldrich), K-Ras (1 mg/mL, Thermo Fisher Scientific), p-B-Raf (1 mg/mL, Sigma-Aldrich), p-MEK (~1 mg/mL, Invitrogen), MEK (~1 mg/mL, Invitrogen), p-ERK (0.5 mg/mL, Invitrogen), ERK (0.5 mg/mL, Invitrogen), p-mTOR (0.5 mg/mL, Invitrogen), mTOR (1 mg/mL, Thermo Fisher Scientific), p-PI3K (1 mg/mL, Invitrogen), PI3K (1 mg/mL, Thermo Fisher Scientific), p-AKT (1 mg/mL, Invitrogen), AKT (0.1 mg/mL, Invitrogen), and GAPDH (0.5 mg/mL, Merck, Darmstadt, Germany). Then, the blots went through incubation with secondary antibody (~2 mg/mL, Sigma-Aldrich). At length, chemiluminescence system supplied by GE Healthcare (Chicago) was utilized for protein detection. The experiment was performed in triplicate.

### 2.14. Statistical Analysis

All the experiments were performed in triplicate. Statistical analysis of experimental data was processed by SPSS software (V22.0). All data were shown as mean ± standard deviation (SD). In addition, Student's *t*-test or one-way ANOVA was applied for comparison of group difference between two or more groups. A *P* value < 0.05 was considered as statistically significant.

## 3. Results

### 3.1. MIR4435-2HG Expression Is Upregulated in BCa and Associated with Poor Survival Outcome

With the application of GEPIA database (http://gepia2.cancer-pku.cn/#index), we found that MIR4435-2HG expression was overtly increased in BCa tissues versus normal tissues (Figure 1(a)). Through RT-qPCR, we examined the expression of MIR4435-2GH in normal cell line SV-HUC-1 and BCa cell lines (T24, HT-1197, HT-1376, and 5637). It was found that MIR4425-2HG was highly expressed in BCa cell lines versus normal cell line (Figure 1(b)). At the same time, survival analysis indicated that high expression of MIR4435-2HG was related to an unfavorable overall survival in patients with BCa (Figure 1(c)). Overall, lncRNA MIR4435-2HG expression is prominently elevated in BCa.

The article "lncRNA MIR4435-2HG Accelerates the Development of Bladder Cancer through Enhancing IQGAP3 and CDCA5 Expression" was retracted in 2024. Reasons: signs of a paper mill; suspected computer-generated content; unreliable results or conclusions; concerns about the data.

### 3.2. MIR4435-2HG Insufficiency Blocks Cell Proliferation, Migration, and Invasion in BCa

To unearth the impact of MIR4435-2HG on BCa progression, we carried out a series of functional experiments. Firstly, MIR4435-2HG was knocked down in T24 and 5637 cells (Figure 2(a)). CCK-8 assay demonstrated that when MIR4435-2HG was silenced, the viability of BCa cells was accordingly inhibited (Figure 2(b)). Also, EdU-positive cells were largely reduced in BCa cells under MIR4435-2HG silencing, which confirmed that MIR4435-2HG depletion hinders cell proliferation (Figure 2(c)). Besides, wound healing and transwell assays were implemented to assess the migratory capacity of BCa cells. MIR4435-2HG deficiency inhibited wound closure and led to the decreased number of migrated cells (Figures 2(d) and 2(e)). The results turned out that silencing of MIR4435-2HG markedly attenuated the migratory capacity of T24 and 5637 cells. Similarly, we found a distinct decrease in number of invaded cells caused by deficiency of MIR4435-2HG (Figure 2(f)). To summarize, MIR4435-2HG aggravates cell proliferation, migration, and invasion in BCa.

### 3.3. miR-2467-3p Is Sequestered by MIR4435-2HG

We next explored the molecular mechanism underlying MIR4435-2HG-mediated BCa progression. Firstly, we conducted cytoplasmic-nuclear fractionation and FISH assays to detect the distribution of MIR4435-2HG in BCa cells. The results presented that MIR4435-2HG was primarily accumulated in the cytoplasm (Figures 3(a) and 3(b)), which suggested that MIR4435-2HG might exert function at the posttranscriptional level in BCa cells. RIP assay proved that MIR4435-2HG was highly abundant in Ago2-bound complex (Figure 3(c)), which suggested that MIR4435-2HG might serve as a miRNA sponge in an Ago2-dependent manner. With the help of starBase website (http://starbase.sysu.edu.cn/index.php) (CLIP Data ≥ 5), we predicted 17 potential miRNAs. RNA pull-down assay further verified that only miR-2467-3p was observably enriched in the complexes pulled down by biotinylated MIR4435-2HG probe (Figure 3(d)). As demonstrated in Figure 3(e), miR-2467-3p expression was prominently downregulated in BCa cell lines versus normal cell line. The predicted binding sequences between MIR4435-2HG and miR-2467-3p are displayed in Figure 3(f). Subsequently, miR-2467-3p expression was enhanced in BCa cells after transfection of miR-2467-3p mimics (Figure 3(g)). Then, luciferase reporter assay was performed to detect the binding between MIR4435-2HG and miR-2467-3p. We found that miR-2467-3p upregulation significantly reduced the luciferase activity of MIR4435-2HG-Wt versus the control group (Figure 3(h)). In a word, MIR4435-2HG functions as a ceRNA against miR-2467-3p.

The article "lncRNA MIR4435-2HG Accelerates the Development of Bladder Cancer through Enhancing IQGAP3 and CDCA5 Expression" was retracted in 2024. Reasons: signs of a paper mill; suspected computer-generated content; unreliable results or conclusions; concerns about the data.

### 3.4. IQGAP3 and CDCA5 Are Downstream Genes of miR-2467-3p

Further, we investigated the downstream target of miR-2467-3p. By means of GEPIA and starBase, overlap of Venn diagram exhibited 2 potential mRNAs (Figure 4(a)). RT-qPCR analysis revealed that IQGAP3 and CDCA5 levels were both decreased in BCa cells under miR-2467-3p overexpression (Figure 4(b)). Hence, we speculated that IQGAP3 and CDCA5 were downstream targets of miR-2467-3p. The binding sites between miR-2467-3p and IQGAP3 or CDCA5 are exhibited in Figure 4(c). RIP assay manifested that MIR4435-2HG, miR-2467-3p, IQGAP3, and CDCA5 were highly abundant in the complex bound with Ago2 antibody (Figure 4(d)), verifying that miR-2467-3p binds to IQGAP3 and CDCA5. Luciferase reporter assays also validated the binding between miR-2467-3p and IQGAP3 or CDCA5 (Figure 4(e)). The level of miR-2467-3p was reduced in miR-2467-3p-deficient T24 and 5637 cells (Figure 4(f)). In addition, MIR4435-2HG deficiency caused a distinct reduction in the expression of IQGAP3 and CDCA5 at mRNA level and protein level while this effect was fully restored by miR-2467-3p silencing (Figures 4(g) and 4(h)). Taken together, miR-2467-3p targets IQGAP3 and CDCA5 and negatively regulates their expression.

### 3.5. IQGAP3 Activates the Ras/Raf/MEK/ERK Signaling Pathway and CDCA5 Stimulates the PI3K/AKT/mTOR Signaling Pathway

IQGAP3 and CDCA5 have been reported to be involved in the Ras/Raf/MEK/ERK and PI3K/AKT/mTOR pathways, respectively, [27, 28]. Thereafter, we conducted western blot analysis to validate whether IQGAP3 and CDCA5 influence key factors in the related signaling pathways. First of all, IQGAP3 expression was decreased in T24 and 5637 cells (Figure 5(a)). Western blot analyzed that EGFR, k-Ras, p-B-Raf, p-MEK, and p-ERK protein levels were all lessened in IQGAP3-inhibited BCa cells (Figure 5(b)). Meanwhile, CDCA5 was also knocked down in T24 and 5637 cells (Figure 5(c)). Likewise, the expression of p-mTOR, p-PI3K, and p-AKT at protein level was also decreased in BCa cells on account of CDCA5 abrogation (Figure 5(d)). Altogether, IQGAP3 and CDCA5 are important activators of the Ras/Raf/MEK/ERK and PI3K/AKT/mTOR pathways, respectively.

### 3.6. MIR4435-2HG Contributes to BCa Progression via Modulation of the miR-2467-3p/IQGAP3/CDCA5 Axis

To verify the role of the MIR4435-2HG/miR-2467-3p/IQGAP3/CDCA5 axis in BCa, we performed a list of rescue experiments. The expression levels of IQGAP3 and CDCA5 were greatly elevated in T24 cells after transfection of pcDNA3.1/IQGAP3 and pcDNA3.1/CDCA5 (Figure 6(a)). As shown in CCK-8 and EdU assays, MIR4435-2HG interference resulted in a decrease on cell proliferation while this suppression effect was thoroughly restored by miR-2467-3p silencing and partially altered by overexpression of either IQGAP3 or CDCA5 (Figures 6(b) and 6(c)). In like manner, wound healing and transwell assays elucidated that miR-2467-3p inhibition completely offset the suppressive effect of MIR4435-2HG inhibition on cell migration and invasion, whereas either IQGAP3 overexpression or CDCA5 overexpression partially countervailed the impaired cell migration and invasion imposed by deletion of MIR4435-2HG (Figures 6(d)–6(f)). All in all, MIR4435-2HG stimulates the progression of BCa via targeting the miR-2467-3p/IQGAP3 or miR-2467-3p/CDCA5 axis.

The article "lncRNA MIR4435-2HG Accelerates the Development of Bladder Cancer through Enhancing IQGAP3 and CDCA5 Expression" was retracted in 2024. Reasons: signs of a paper mill; suspected computer-generated content; unreliable results or conclusions; concerns about the data.

## 4. Discussion

Emerging evidence has highlighted that lncRNA MIR4435-2HG influences the malignant phenotypes of cancer cells. For example, Kong et al. have unmasked that MIR4435-2HG boosts cell proliferation in hepatocellular carcinoma through enhancing miR-487a expression [16]. Yang et al. have manifested that MIR4435-2HG targets the miR-206/YAP1 axis to advance colorectal cancer cell proliferation and metastasis [29]. Liu et al. have disclosed that MIR4435-2HG suppresses the process of osteoarthritis via binding to miR-510-3p [30]. In this research, we demonstrated that MIR4435-2HG expression was obviously high in BCa cells and associated with poor survival in BCa patients. Moreover, our study firstly identified the oncogenic role and molecular mechanism of MIR4435-2HG in BCa. Specifically, we found that downregulation of MIR4435-2HG impairs the proliferative, migratory, and invasive abilities of BCa cells.

The lncRNA-miRNA-mRNA ceRNA network has been regarded to be critical in BCa pathogenesis [31, 32]. Here, the present study indicated that MIR4435-2HG might serve as a ceRNA to participate in posttranscriptional events. Importantly, miR-2467-3p was validated to be a downstream target of MIR4435-2HG.

Besides, miR-2467-3p suppresses the progression of colorectal cancer, cervical cancer, and non-small-cell lung cancer [33–35]. Consistent with these findings, our study manifested that miR-2467-3p expression was downregulated in BCa cells. More importantly, miR-2467-3p was verified to participate in the regulation of BCa progression.

IQGAP3 has been shown to govern cell proliferation and migration [36] and has been certified to exhibit high expression in some cancers, such as breast cancer, lung cancer, prostate cancer, kidney cancer, liver cancer, and colorectal cancer [37]. Also, previous studies have demonstrated the oncogenic functions of IQGAP3 in cancers, such as ovarian cancer [38] and gastric cancer [39]. Besides, IQGAP3 urinary cell-free NA may be utilized as a new noninvasive bladder cancer diagnostic marker [40]. Additionally, IQGAP3 can interact with ERK1 to modulate the Ras/Raf/MEK/ERK signaling pathway [27]. Moreover, CDCA5 has been confirmed to aggravate cell cycle and inhibit cell apoptosis in BCa via activation of the PI3K/AKT/mTOR signaling pathway [28]. Through our investigation, IQGAP3 and CDCA5 were found to be targeted by miR-2467-3p and negatively regulated by miR-2467-3p in BCa. More interestingly, downregulation of IQGAP3 or CDCA5 inactivates the MEK/ERK pathway and PI3K/AKT/mTOR pathway, respectively. In this research, we found that the MIR4435-2HG/miR-2467-3p/IQGAP3/CDCA5 axis enhances BCa progression.

The article "lncRNA MIR4435-2HG Accelerates the Development of Bladder Cancer through Enhancing IQGAP3 and CDCA5 Expression" was retracted in 2024. Reasons: signs of a paper mill; suspected computer-generated content; unreliable results or conclusions; concerns about the data.

All in all, MIR4435-2HG was demonstrated to be an oncogene in BCa and predicted poor survival outcome. Deficiency of MIR4435-2HG repressed BCa cell proliferation, migration, and invasion. As for the underlying mechanism, MIR4435-2HG sequestered miR-2467-3p to modulate the expression of IQGAP3 and CDCA5 via ceRNA mode, leading to activation of the MEK/ERK and PI3K/AKT/mTOR pathways. All the findings might provide novel insights for BCa treatment.

## Figures and Tables

**Figure 1:** MIR4435-2HG expression is upregulated in BCa and associated with poor survival outcome. (a) GEPIA of MIR4435-2HG expression in BCa samples (*n* = 404) and normal samples (*n* = 28). (b) RT-qPCR detected MIR4435-2HG expression in normal cell line (SV-HUC-1) and BCa cell lines (T24, HT-1197, HT-1376, and 5637). (c) GEPIA correlation analysis of MIR4435-2HG expression and overall survival rate of BCa patients. ^∗^*P* < 0.05; ^∗∗^*P* < 0.01.

**Figure 2:** MIR4435-2HG insufficiency blocks cell proliferation, migration, and invasion in BCa. (a) Gene ablation of MIR4435-2HG in MIR4435-2HG-deficient T24 and 5637 cells was tested via RT-qPCR. (b, c) CCK-8 and EdU assays (magnification × 100) were used to evaluate cell proliferation. (d–f) Wound healing (magnification × 100) and transwell assays (magnification × 100) were used to determine the migratory and invasive capacities of BCa cells. ^∗∗^*P* < 0.01.

**Figure 3:** miR-2467-3p is sequestered by MIR4435-2HG. (a, b) Subcellular fractionation and FISH assays (magnification × 1,000) were conducted to explore the distribution of MIR4435-2HG in BCa cells. (c) RIP assay examined the enrichment of MIR4435-2HG in Ago2-RISC. (d) The enrichment of predicted 17 miRNAs in the complexes pulled down by biotinylated MIR4435-2HG probe was measured by RNA pull-down assay. (e) RT-qPCR examined the expression of miR-2467-3p in BCa cell lines and SV-HUC-1. (f) The starBase website was applied to predict the binding sites between MIR4435-2HG and miR-2467-3p. (g) Gene overexpression efficiency of miR-2467-3p was verified by RT-qPCR. (h) The physical interaction between MIR4435-2HG and miR-2467-3p was detected by luciferase reporter assay. ^∗^*P* < 0.05; ^∗∗^*P* < 0.01.

The article "lncRNA MIR4435-2HG Accelerates the Development of Bladder Cancer through Enhancing IQGAP3 and CDCA5 Expression" was retracted in 2024. Reasons: signs of a paper mill; suspected computer-generated content; unreliable results or conclusions; concerns about the data.

**Figure 4:** IQGAP3 and CDCA5 are downstream genes of miR-2467-3p. (a) Overlap of Venn diagram exhibited 2 predicted mRNAs. (b) IQGAP3 and CDCA5 levels were detected in miR-2467-3p-overexpressing BCa cells. (c) The predicted binding regions between miR-2467-3p and IQGAP3 or CDCA5. (d) The relationship among MIR4435-2HG, miR-2467-3p, IQGAP3, and CDCA5 was detected by RIP assay. (e) Luciferase activity in the IQGAP3 3′UTR-Wt group, IQGAP3 3′UTR-Mut group, CDCA5 3′UTR-Wt group, and CDCA5 3′UTR-Mut group in BCa cells cotransfected with miR-2467-3pmimics was detected. (f) Transfection of miR-2467-3p inhibitor into BCa cells was performed for miR-2467-3p silencing. (g, h) The expression of IQGAP3 and CDCA5 at mRNA level and protein level was detected in different groups. ^∗∗^*P* < 0.01.

**Figure 5:** IQGAP3 activates the Ras/Raf/MEK/ERK signaling pathway, and CDCA5 stimulates the PI3K/AKT/mTOR signaling pathway. (a) Gene deletion efficiency of IQGAP3 in T24 and 5637 cells was examined by RT-qPCR. (b) Western blot analyzed the protein levels of EGFR, K-Ras, p-B-Raf, p-MEK, MEK, p-ERK, and ERK in IQGAP3-deficient BCa cells. (c) Gene deletion efficiency of CDCA5 in BCa cells was assessed via RT-qPCR. (d) The levels of PI3K/AKT/mTOR signaling pathway-associated proteins in CDCA5-silenced BCa cells were analyzed via western blot. ^∗∗^*P* < 0.01.

**Figure 6:** MIR4435-2HG contributes to BCa progression via modulation of the miR-2467-3p/IQGAP3/CDCA5 axis. (a) Gene upregulation efficiency of IQGAP3 and CDCA5 in T24 cells was tested via RT-qPCR. (b, c) CCK-8 and EdU assays (magnification × 100) were conducted to detect the proliferation of T24 cells under different transfections. (d–f) The migration and invasion capacities of BCa cells under different transfections were assessed by wound healing (magnification × 100) and transwell assays (magnification × 100). ^∗^*P* < 0.05; ^∗∗^*P* < 0.01.

## Data Availability

The data used to support the findings of this study are included within the article.

## Supplementary Materials

Supplementary Materials Supplementary Table 1: specific primers used for RT-qPCR. F: forward; R: reverse.
